The article "Business English Translation Model Based on BP Neural Network Optimized by Genetic Algorithm" was retracted in 2023. Reasons: suspected computer-generated content; unreliable results or conclusions; concerns about the data; concerns about the results or conclusions.

# Business English Translation Model Based on BP Neural Network Optimized by Genetic Algorithm

**DOI:** 10.1155/2021/2837584

**Published:** 2021-08-10

**Authors:** Yanning Chen

**Affiliations:** School of International Studies, Hunan Institute of Technology, Hengyang 421002, China

## Abstract

In recent years, most of the communication places are using business English manual simultaneous interpretation or electronic equipment translation. In the context of diverse cultures, the way English is used and its grammar vary from country to country. In the face of this situation, how to optimize business English translation technology and improve the accuracy of business communication content is one of the research contents of scholars all over the world. This paper first introduces the purpose of business English translation and the gap between business English translation and general English translation. Secondly, a genetic algorithm is used to optimize the structure of the BP neural network, and the combination of the two improves the ability of translation search. This paper compares the influence of the traditional BP algorithm and the BP algorithm optimized by genetic algorithm on the construction of a business English translation model. The results show that BP neural network optimized by the genetic algorithm can improve the speed of business English text translation, reduce the impact of semantic errors on the accuracy of the translation model, and improve the efficiency of translation.

## 1. Introduction

With the development of globalization in various fields, business English has become more widely used. With the frequent use of business English, the requirements for translation in business activities are becoming more and more strict. As a global communication language, business English includes a lot of professional terminology knowledge in addition to everyday language. Therefore, there are great differences between business English and general English translation [1]. Due to the high professional requirements of business English, the requirements of skills and efficiency in the process of translation are also higher. As a kind of English translation, we need to study how to be more suitable for effective communication in the business environment. In the process of business English translation, we often encounter communication difficulties due to the differences in the use of national languages, different daily expressions, different traditional cultural vocabulary, and so on. In order to have better language communication, we need to solve the conflict problem caused by cultural differences [2].

According to the BP neural network training model, in the process of model building, efficient learning training content can make translation reduce unnecessary time [3]. First of all, in the process of model building, we need to manually record the scope of cultural differences to better analyze the differences and according to the current environment to solve the problem of translation. Secondly, we need to show the professional ability of business and effectively distinguish the differences between business and general English translation [4]. In the expression of translation sentences, the optimized simple language is used for elaboration, and the simplified language can be used for effective communication [5]. In the process of using simplified sentences to express the complete meaning, we need to ensure the accuracy and real-time of the whole translation. Finally, the rules of primary and secondary sentences in the process of business English translation need to ensure the smoothness of translation sentences and the relationship between primary and secondary sentences.

Business English can be divided into two parts: business and English. It is composed of ordinary English structure, according to the grammatical rules of ordinary English, the scope of words, and the relationship between primary and secondary business English. In addition to including business professional knowledge vocabulary and basic vocabulary, the purpose of use has also changed. It is mainly used in business services and information transmission, and the use standards are more stringent [6]. Before the translation work, it is necessary to master the language usage of different cultural differences [7]. English is an international language. The grammar and meaning of English words are different in different regions. For example, American English and British English have different pronunciations, conjunctions, and tones [8]. In business activities, due to the cultural collision of different countries, there are many different cultural translations of the same thing. When cultural differences occur in translation, the details of communication cannot be consistent [9]. In order to better promote communication, we need to bring ourselves into the translation process. Business English is not only a service-oriented language but also a competitive language. Therefore, the expression of language is more direct and clear. We need to express our purpose in the shortest possible time to avoid the economic loss caused by the waste of time [10]. In addition to direct mood and context, objectivity should also be ensured in the form of expression. Translators should not include subjective emotional opinions but should try their best to maintain an objective attitude, so as to maintain a professional and rigorous image in the process of business English translation [11].

In the process of business English translation model construction, BP neural network algorithm can be used. According to the data collected by the neural network algorithm, the range can be expanded to several times the effect of the ordinary algorithm. Due to a large amount of data, it can reflect the speed and accuracy of the translation process [12]. The basic models are regression models, such as the empirical regression model and the logical regression model. Time comparison and accuracy of translators are selected as the basic variables of the model, and the model is simulated through the relationship between the data [13]. The regression model based on the time series and variable data of the LSTM neural network algorithm can predict the effect and time accuracy of business English translation [14]. Regression models include linear and nonlinear models. The neural network is nonlinear based on traditional manual use. Through the learning and training function to remodel the model, the purpose of approaching any nonlinear contrast function can be achieved, and the prediction results can still maintain the accuracy in the case of less data sources [15]. Finally, in the process of business English translation model establishment and prediction function construction, it can improve the calculation speed and reduce unnecessary waste of time. Under the influence of neural network algorithm layer control and weight ratio, the training time algorithm has great convergence ability [16]. In order to solve the problem of complex model structure in the process of translation training, this paper proposes a structure optimization method of BP neural network based on a genetic algorithm. By controlling the number of data sources, the number of hidden layers of the neural network before and after optimization was compared [17] so as to improve the overall performance of the model and improve the time usage.

This paper studies the construction process of a business English translation model based on a neural network algorithm. The BP neural network algorithm is compared with the traditional neural network algorithm, and the genetic algorithm is used to optimize the BP neural network algorithm model. The purpose of this study is to predict the translation function of business English. This paper mainly studies the optimization method of genetic algorithm to improve the structure of BP neural network, selects particle swarm optimization algorithm to build the translation model in the traditional neural algorithm, and puts forward the optimal effect form of business English translation. Finally, the learning effect of the model is analyzed from the experimental results and operation process of the constructed neural network algorithm and particle swarm optimization algorithm model, which helps to improve the overall performance and work level of business English translation.

## 2. A Study on the Translation Technology of Business English Based on Genetic Algorithm Optimization of BP Neural Network

### 2.1. Research on BP Neural Network Structure Technology Based on Genetic Algorithm Optimization

Particle swarm optimization (PSO) has been widely used in many fields, such as function optimization, image processing, and geodesy. With the expansion of its application, the PSO algorithm has some problems, such as premature convergence, dimension disaster, and easy to fall into local extremum. The genetic algorithm belongs to evolutionary computing, which is an intelligent algorithm with the development of artificial intelligence. As its name suggests, genetic algorithms are inspired by Darwin's theory of evolution. In short, it is a method to search for the optimal solution by simulating the natural evolution process. In addition, pattern search technology, fractional particle swarm optimization, backtracking search optimization, fireworks, and many other optimization algorithms also have the characteristics of searching for the optimal solution. The BP neural network optimized by the genetic algorithm proposed in this study can improve the optimization speed, reduce the influence of model accuracy, and improve the calculation efficiency.

In order to solve the problem of complex training caused by the multilayer structure of neural network algorithm in the training process, we propose the method of using a genetic algorithm to optimize the structure of the neural network [18]. With the trend that artificial neural networks can gradually solve complex problems and is difficult to define problems, this algorithm has been applied to intelligent equipment, robot simulation, computer recognition, information data processing, and other fields [19]. Artificial neural networks can learn logic through self-training without determining the relationship between variables. The algorithm is developed and used through intelligent data processing [20]. In BP neural network through error inversion in the multilevel feedback network structure, using a recursive algorithm to gradually optimize the actual data, the output error square is the minimum [21]. If the structure of the artificial neural network is too complex, it will lead to a large difference in the output results; on the contrary, it will lead to a low learning and training ability. How to quickly and accurately improve the structure of the neural network has always been the focus of attention of scholars all over the world [22].

BP neural network contrast propagation is divided into multilevel, mainly including input, output, and fading layers. The structure of the BP network is shown in Figure 1.

It can be seen from the figure that the input layer and the output layer have multivariable element data, respectively, and the related variables among the three layers are weight and threshold. It also includes unknown variables expected for the output layer. According to the screening principle, the genetic algorithm selects the appropriate path to remove the complex path, which is a natural algorithm to simulate the evolution process. It is an algorithm to find the maximum probability and the optimal solution in the process of global variable prediction training. The core of the algorithm is to find the optimal solution and calculate the optimal probability. In the interaction process of genetic algorithm, the crossover and fusion between individual variables and population variables, individual variables, and individuals are carried out, and the most suitable combination variants are selected. The new variant is more suitable for the expected data than the original data. A new output variable value is formed after several cycles of output. The structure of the BP neural network optimized by the genetic algorithm is shown in Figure 2.

The weight variables and threshold variables of the initial value of the basic BP neural network are random numbers in a small range, which need to be superimposed many times in the process of updating the network structure. The global optimal solution and probability can be obtained by a genetic algorithm. Therefore, the genetic algorithm used in the figure to optimize the initial value of the BP neural network can improve the efficiency of learning and training and the speed of computing data results. The genetic algorithm encodes the data source and sets the error function

(1) $$\begin{array}{c} F=k\left(\sum_{j=1}^{n}\text{abs}\left(y_{j}-o_{j}\right)\right). \end{array}$$

In equation (1), *y*_*j*_ is the expected value of network nodes, *o*_*j*_ is the expected output value of network nodes, *n* is the number of network nodes, and *k* is the structural adjustment variable. The fitness value is calculated according to the formula to judge the weight and threshold after optimization. If the conditions meet, it is added to the calculation of the neural network error formula. The formula is as follows:

(2) $$\begin{array}{c} E\left(\omega ,b\right)=\frac{1}{2}\sum_{j=0}^{n-1}{\left(y_{j}-o_{j}\right)}^{2}. \end{array}$$

In equation (2), the difference between the output variables of each node and the expected variables is summed by square root, and then half of the calculation result is regarded as the network error variable. When the network algorithm model performs a multilevel calculation process and meets the specified accuracy, the calculation process is stopped and the training results are output. Then, according to the SIM function, the simulation results are obtained.

The input and output layers of multilayer neural network structure are embedded in a gradually hidden layer, and the unit nerves in the same layer are not related to each other. The display form is that the unit nerve is connected with the next layer, and the structure is shown in Figure 3.

It can be seen from the figure that the unit nerves of each level of the multilayer neural network structure are independent of each other, and the input layer and output layer are added with the gradually hidden layer structure, which can connect the independent unit nerves with the up and down.

The operation of the artificial neural network is the process of solving input and output variables by using a nonlinear function. The basic unit is the neural unit, as well as data elements. The actual results are measured according to the input data source, and the data is output to the construction model in order to help the learning and training process. When the structure of the training neural network is formed, it is necessary to assign weights according to the path of each unit. Each group of data source input calculation results as output variables, and the experimental data of the control group need to reach a certain similar value. The neural units of multilevel are connected with each other, and the weight value is input into the neural unit to calculate the sum. The output data is adjusted according to the activation function. The function formula is as follows:

(3) $$\begin{array}{c} f\left(x\right)=\frac{1}{1+e^{-x}}. \end{array}$$

In the variable of the gradually hidden layer, each variable represents the number of neural units, and the output variable of neural units is calculated according to the following formula:

(4) $$\begin{array}{c} h_{i}^{j}=f\left(\sum_{k=n}^{n_{i-1}}w_{k,j}^{i-1}h_{i-1}^{k}\right),\;i=2,\ldots ,N,\;j=1,\ldots ,n_{i}. \end{array}$$

Among them, *w*_*k*,*j*_^*i*^ represents the weight between different levels of the unit nerves in the gradually hidden layer, *n*_*i*_ represents the number of unit nerves in the *i*^th^ gradually hidden layer, and the output variable of the *i*^th^ layer is calculated by the following formula:

(5) $$\begin{array}{c} h_{i}=\left(h_{i}^{1},h_{i}^{2},\ldots ,h_{i}^{ni}\right). \end{array}$$

The unit nerve in the output layer can get the fading output results of other layers:

(6) $$\begin{array}{c} \left\{\begin{array}{c} y_{i}=f\left(\sum_{k=1}^{n_{N}}w^{N}k,jh_{N}^{k}\right),\\ Y=\left(y_{1,\ldots ,}y_{j,\ldots ,}y_{m}\right)=F\left(w,x\right), \end{array}\right) \end{array}$$

where *Y*=(*y*_1,…,_*y*_*j*,…,_*y*_*m*_) is the output variable and *F* is the transfer function; the definition formula of weight matrix is as follows:

(7) $$\begin{array}{c} W=\left[W^{0},\ldots ,W^{i},\ldots ,W^{N}\right]. \end{array}$$

In order to optimize the structure of the BP neural network, the new calculation formula is changed accordingly. The calculation formula is as follows:

(8) $$\begin{array}{c} F\left(U,W,X\right)=Y=\left(y_{1},y_{2},\ldots ,y_{n_{N+1}}\right). \end{array}$$

The value of the vector is 0 or 1. The output value of the first fading layer can be calculated by the following formula:

(9) $$\begin{array}{c} h_{1}=\left(\begin{array}{c} h_{1}^{i}\\ h_{1}^{j}\\ h_{1}^{ni} \end{array}\right)=\left(\begin{array}{c} f\left(\sum_{k=1}^{n_{0}}w_{k,i}^{0}x_{k}\right)\\ f\left(\sum_{k=1}^{n_{0}}w_{k,j}^{0}x_{k}\right)\\ f\left(\sum_{k=1}^{n_{0}}w_{k,n_{1}}^{0}x_{k}\right) \end{array}\right). \end{array}$$

Among them, (*x*_1_, *x*_2_,…, *x*_*n*0_) represents the input data neural unit, and the output formula of gradually hidden level calculation is as follows:

(10) $$\begin{array}{c} h_{1}=\left(1-u_{i-1}\right)h_{i-1}+u_{i-1}\left(\begin{array}{c} f\left(\sum_{k=1}^{n_{i-1}}w_{k,i}^{i-1}h_{i-1}^{k}\right)\\ f\left(\sum_{k=1}^{n_{i-1}}w_{k,j}^{i-1}h_{i-1}^{k}\right)\\ f\left(\sum_{k=1}^{n_{i-1}}w_{k,n_{1}}^{i-1}h_{i-1}^{k}\right) \end{array}\right),\\ h_{N}=\left(1-u_{N-1}\right)h_{N-1}+u_{N-1}\left(\begin{array}{c} f\left(\sum_{k=1}^{n_{N-1}}w_{k,i}^{N-1}h_{N-1}^{k}\right)\\ f\left(\sum_{k=1}^{n_{N-1}}w_{k,j}^{N-1}h_{N-1}^{k}\right)\\ f\left(\sum_{k=1}^{n_{N-1}}w_{k,n_{N}}^{N-1}h_{N-1}^{k}\right) \end{array}\right). \end{array}$$

The final output formula of the optimized neural unit is as follows:

(11) $$\begin{array}{c} y_{j=}f\left(\sum_{k=1}^{n_{N}}w_{k,j}^{N}h_{N}^{k}\right),\;j=1,\ldots ,n_{N+1}. \end{array}$$

The error formula between the input and output of the optimized objective function programming model and the expected results is as follows:

(12) $$\begin{array}{c} {\left\|F\left(U,X,W\right)-d\right\|}^{2},\\ \underset{i=1,\ldots ,N-1}{\sum }u_{i}\geq 1. \end{array}$$

Through the above formula, the traditional BP neural network is optimized to form the optimized neural network structure matrix. This matrix adopts nonlinear function programming to study the optimization of the BP neural network by genetic algorithm. Before getting the output result of the hidden layer optimization, the vector is reassigned to get the latest output data. The latest data is taken as the model calculation variables of the objective function, and whether the optimized model error value meets the requirements is analyzed. In the process of optimizing BP neural network structure by genetic algorithm, the model of solving nonlinear variables is constructed according to the rules of the GA algorithm. Different variables and variation rules are selected as the benchmark. Each data solution represents the coded chromosome, and the chromosome represents the variable value. Then, the optimal individuals are selected according to a fixed number of variable populations to split. Finally, the stacking times of the maximum range are achieved. The initial random generation of an unknown number of structural data is achieved, according to the structure of a new individual. The number of individuals is unknown. Variable parameters are set according to the range they can hold. The calculation process between layers is shown in Figure 4.

Fitness is generated in the process of individual exchange, which is used to measure the individual advantage and best fit data in group variables. Fitness is used as the judgment basis of feature point combination. The value of the individual variable is selected according to the fitness of numerical matching. This process depends on the value of the variable calculation function. The larger the fitness degree, the more obvious the matching trend among individuals. The fitness formula is as follows:

(13) $$\begin{array}{c} \text{Fitness}\left(i\right)=M-\text{objctive}\left(i\right). \end{array}$$

In the fitness matching selection, we can select suitable individuals for the model. The objective function is constructed according to the model, which is used to build the translation model and predict the results. It is equivalent to selecting the optimal solution from the global variables, according to this proportion method to get the best data value of the prediction model.

### 2.2. Research on the Establishment of Business English Translation Model Based on Neural Network Algorithm

Under the premise of the continuous development of computer machine translation, we find that there are many problems. In view of the above problems, we need to pay attention to the theoretical model of unified MT in-depth learning. And the construction of the connection between the endpoints of the neural network structure needs to be optimized. Former researchers have built the encoder and decoder in the machine construction of the end-to-end model [23, 24]. They realized the assumption of probability model construction in language translation. The language content of source data acquisition is coded and mapped to form calculation variables. Finally, the final transformation meaning of target variables is obtained according to the decoding process. The coding model is built according to CNN convolutional neural network, and the decoding model is constructed by a recursive algorithm, so as to achieve the historical data and processed data series [25]. We build a business English translation model based on the neural network optimization algorithm. In the process of language, statement, and semantic classification, the neural network has a key effect. But the effect is far from that of the human brain. It can not think about the complicated problems and make up the related logical sequence as the human brain. With the complexity of data acquisition and time series, the solution is intelligent based on the recursive algorithm in the neural network.

The conversion mechanism is based on the feedforward network structure without the closed-loop process. That is, it is similar to the BP neural network model optimized by a genetic algorithm. Variables are selected instead of input data, output, and fade data. The weight matrix and threshold range are calculated. The specific process is as follows:

(14) $$\begin{array}{c} \left\{\begin{array}{c} r_{1}=Uv_{1}+Mh_{0},\\ h_{1}=f\left(r_{1}\right),\\ w_{1}=g\left(Nh_{1}\right), \end{array}\right) \end{array}$$

where *f* and *g* are activation functions. In the process of time series, the storage state of each time is the data input value of the next activity. The formula is as follows:

(15) $$\begin{array}{c} \left\{\begin{array}{c} r_{2}=Uv_{2}+Mh_{1},\\ h_{2}=f\left(r_{2}\right),\\ w_{2}=g\left(Nh_{2}\right). \end{array}\right) \end{array}$$

The specific state formula of the target time is as follows:

(16) $$\begin{array}{c} \left\{\begin{array}{c} r_{k}=Uv_{k}+Mh_{k},\\ h_{k}=f\left(r_{k}\right),\\ w_{k}=g\left(Nh_{k}\right). \end{array}\right) \end{array}$$

From the above structure formula, it can be seen that the recursive algorithm is prone to the loss of hours in the neural network training model. This will lead to the fact that the training process can not be normal operation and continuous. We set the threshold and gradient range of the overall benchmark to ensure the operation of the algorithm. When the threshold value exceeds the set range, intercept processing is taken immediately. In the structure of the artificial neural network, there are many units and nodes. Multilayer neural network structure is the most widely used. Multilayer structure and single neural network are input-output and gradually hidden layer as the basic structural framework. The process of processing information is similar. In the process of business English translation, it is very necessary to analyze the patterns according to the collected data sets and get accurate results. Therefore, a learning and training model is set up to analyze the translation process. The structure of the analysis model is shown in Figure 5.

According to the learning ability model, this paper analyzes the characteristics in the process of business English translation training. The data value in the process of business English translation training is obtained as an index for training translation ability. In the process of initial data collection, a sampling survey and questionnaire can be used. Then, the data source extraction process is carried out, and the interference data that has no effect on the data set calculation is deleted according to the information processing preprocessing. In the process of calculation, due to the omission and dissatisfaction of data, there is no need to require too much for the comparison value of standard results. Then, the preprocessed data is analyzed by neural network structure to determine the network model structure and the number of layers:

(17) $$\begin{array}{c} J=\sqrt{\text{MN}}. \end{array}$$

In the formula, *J* represents the nodes of the gradually hidden layer, and MN represents the number of output and input nodes. According to the calculation, the relationship curve between the training analysis value and each layer node can be obtained. After simplifying the relationship curve, we can get the change of the structure times of the whole training model. The expected node and training times curve and the actual result curve are shown in Figure 6.

It can be seen from Figure 7 that the more the number of nodes in the neural network structure appears between multiple levels, the less training and learning times of the whole translation model. In other words, the optimized neural network structure is conducive to the construction of a business English translation model.

## 3. Analysis of Business English Translation Model Based on BP Neural Network Optimized by Genetic Algorithm

### 3.1. Result Analysis of Neural Network Model Optimized by Genetic Algorithm

In the structure of the BP neural network, input, output, and fading are the key contents of the model. According to the continuous property and category property of the data source, there are obvious characteristics such as scattered and disordered rules in the classification. In data classification, we can see that the data set is continuous and regular, so we can solve the problem of feature point distribution in classification according to the coding principle. The number of input layer nodes is still determined by its own characteristic points, and the data of each layer is an unknown number of neuron units. The output layer is the final target variable, and the output neuron value is the final training prediction result. Gradually hidden layer plays the role of connecting the whole neural network structure, as one of the essential links to connect the upper and lower layers. We need to determine the number of nodes and the number of distribution of the gradually hidden layer and carry out the numerical query of neurons according to the characteristics of the whole layer. In the optimization process, the three-layer neural network structure is still used, and the coding formula is used to define variables. The code length formula is as follows:

(18) $$\begin{array}{c} L=nm+ml+m+l. \end{array}$$

In addition to defining the encoding length, in order to analyze the validity of the resulting model, the variables of prediction value, total value, and error analysis were defined. The test results of neural network structure optimized by the genetic algorithm are shown in Table 1.

According to Table 1, according to different artificial neural network structures, the neural network optimized by the algorithm can provide help for the optimal strategy of business English translation. Compared with the traditional neural network structure, the number of the optimal input, output, and fading layer variables after optimization is reduced by three percentage points. When the average RMSE index is less than 1, it can be concluded that the optimized neural network algorithm has a positive and effective impact on the construction of the overall translation model.

### 3.2. Application of Optimized Neural Network Algorithm in Business English Translation Model Construction

Business English translation model based on the concept of structural optimization is improved to achieve efficient structural components and to be able to distinguish professional knowledge from general knowledge in the process of the English translation. In the process of training and learning, the relationship analysis method is used for training. Appropriate variables are selected to represent the statements and syntax rules to reflect the important components of the whole model. The specific framework of the business English translation model is shown in Figure 7.

The process of data preprocessing includes the selection of single syntax and double syntax, short sentences, and long sentences. The neural network structure formed by training is used to generate variable statements, which are used as the data model of BP neural network training. In the process of training, there are corresponding requirements for encoder and decoder. We need to get the data source through the recurrent neural network to assign the variable and then get the semantic expression. According to the monolingual and bilingual compiler, the multilevel gradual time serialization training is adopted, and then, the whole network structure is contacted for translation.

The concept of neural network structure in translation experiment design is the connection between endpoints. In order to improve machine learning, a neural network model is used to train natural language. We use probabilistic translation to build the model, preprocess the source data sentences as a group, and use a neural network to directly affect the function of language translation. The translation model after encoding and decoding is shown in Figure 8 .

In order to compare the influence of semantic feature points on the translation model, we choose the basic path in the study without adding a semantic feature vector and cardinality to build the model. It is concluded that it is similar to the structure of the common translation model, and the nature of language source data is not necessary for the training process. According to the data source, variables are established from left to right, and the former and rear bilingual meanings have similar characteristics. The effect of semantic features on the business English translation model is shown in Figure 9 .

First of all, the features of single and double languages are added, followed by linguistic similarity and semantic ambiguity, and finally sensitivity analysis. The influence of the above variables on the translation model is analyzed by comparing the data indexes. Semantic features have a great influence on the overall translation effect, which shows the importance of semantics in the business English translation model.

## 4. Conclusion

In view of the traditional neural network structure model, this paper proposes a BP neural network structure optimized by a genetic algorithm. Besides genetic algorithm, recursive algorithm and particle swarm optimization algorithm are used to optimize the model. Finally, a BP neural network algorithm suitable for solving complex nonlinear model problems is obtained. After testing, this algorithm can improve the optimal number and weight matrix of each level in the artificial neural network. Compared with the traditional neural network algorithm, the error between the expected output and the calculated value is the smallest. The optimized neural network has a positive impact on the construction of the business English translation model and can meet the needs of the business translation model and process. According to the research results, this paper suggests that, in the construction of the business English translation model, the genetic algorithm is used to optimize the BP neural network technology for business English language generation and semantic translation. This algorithm can improve the traditional neural network algorithm in the construction of the model output accuracy which is not enough.

## Figures and Tables

**Figure 1:** BP network structure chart.

**Figure 2:** Structure chart of BP neural network optimized by genetic algorithm.

**Figure 3:** Structure diagram of multilayer neural network.

**Figure 4:** Calculation process diagram between layers.

**Figure 5:** Analysis model diagram.

**Figure 6:** Graph of node and training times.

**Figure 7:** Business English translation model training framework.

**Figure 8:** Coding and decoding structure model.

**Figure 9:** Influence diagram of semantic business English translation model.

**Table 1:** Test results of neural network structure optimized by genetic algorithm.

Maximum number of iterations	Number of hidden layers	Optimal number of hidden layers	RMSE	Actual times
100	6	4	1.41	19
	10	7	0.86	37

100	8	5	1.02	627
	10	7	0.91	915

10000	8	6	0.73	9433
	10	7	0.78	9043

## Data Availability

The data used to support the findings of this study are available from the corresponding author upon request.
